The article "Multimodal Sentiment Analysis Based on Cross-Modal Attention and Gated Cyclic Hierarchical Fusion Networks" was published in 2022. Journal: Comput Intell Neurosci.

# Multimodal Sentiment Analysis Based on Cross-Modal Attention and Gated Cyclic Hierarchical Fusion Networks

**DOI:** 10.1155/2022/4767437

**Published:** 2022-08-09

**Authors:** Zhibang Quan, Tao Sun, Mengli Su, Jishu Wei

**Affiliations:** School of Computer Science and Technology, Qilu University of Technology (Shandong Academy of Sciences), Jinan 250353, China

## Abstract

Multimodal sentiment analysis has been an active subfield in natural language processing. This makes multimodal sentiment tasks challenging due to the use of different sources for predicting a speaker's sentiment. Previous research has focused on extracting single contextual information within a modality and trying different modality fusion stages to improve prediction accuracy. However, a factor that may lead to poor model performance is that this does not consider the variability between modalities. Furthermore, existing fusion methods tend to extract the representational information of individual modalities before fusion. This ignores the critical role of intermodal interaction information for model prediction. This paper proposes a multimodal sentiment analysis method based on cross-modal attention and gated cyclic hierarchical fusion network MGHF. MGHF is based on the idea of distribution matching, which enables modalities to obtain representational information with a synergistic effect on the overall sentiment orientation in the temporal interaction phase. After that, we designed a gated cyclic hierarchical fusion network that takes text-based acoustic representation, text-based visual representation, and text representation as inputs and eliminates redundant information through a gating mechanism to achieve effective multimodal representation interaction fusion. Our extensive experiments on two publicly available and popular multimodal datasets show that MGHF has significant advantages over previous complex and robust baselines.

## 1. Introduction

Every day, a large and meaningful amount of information is generated around us. Most of this information is generated on the web, and social media is a centralized area of information on the web. It covers many topics, opinions, sentiments, and emotions closely related to our lives. Multimodal sentiment analysis (MSA) has been an active subfield in natural language processing [1, 2]. This is mainly due to its wide range of applications, such as government elections [3], intelligent healthcare [4], and chatbot recommendation systems for human-computer interaction [5]. Compared to traditional sentiment analysis, MSA uses multiple sources (excerpted raw text, acoustic, and visual information) to make predictions about the sentiment expressed by a specific object in a specific period. One of the multimodal sentiment analysis challenges is to model the interactions between different modalities because they contain supplementary and complementary information [6]. Another factor that limits the performance of multimodal sentiment analysis tasks is data fusion. This is because there are multiple recurring problems, such as missing values and misalignment in visual and auditory modalities [7].

In recent years, researchers have designed sophisticated fusion models. Zadeh et al. [8] designed the tensor fusion network, which uses a Cartesian product to fuse the feature vectors of three modalities; this provided a new idea for multimodal data processing. Tsai et al. [9] designed a multimodal transformer that processed all modalities together to obtain the predicted sentiment scores. Although these methods have achieved good results, a problem that may affect the final prediction effect is that these models ignore the differences between different modalities, which may lead to the loss of crucial prediction information during the modal representation acquisition stage. Hazarika et al. [10] designed a modality-specific and modality-invariant feature space, combining two types of representations with similarity loss, reconstruction loss, and dissimilarity loss to evaluate the model effect. Yu et al. [11] used a multitask format and introduced an automatic modal label generation module in the training phase to assist the main task channel, saving manual labelling time, and thus improving efficiency. Although these studies also achieved encouraging results, they lacked intermodal information interaction during the modal fusion phase. Doing so may result in the redundant information present in the upper stage being retained in the final prediction stage, making the model performance poor. As shown in Figure 1, there are two opposite prediction results after the same text interacts with different modalities. For example, an ordinary language with ordinary acoustic features is predicted as a negative sentiment. In contrast, the same type of language with positive visual features is predicted as a positive sentiment. This indicates that different modal combinations have a fundamental impact on sentiment prediction. It should be noted that, in Figure 1, “?” indicates that sentiment cannot be accurately identified, “−” represents negative sentiment, and “+” represents positive sentiment. The number of these symbols signifies the intensity of the sentiment.

To address the mentioned issues, inspired by cross-modal matching and interaction modelling, we propose a novel multimodal sentiment analysis framework, MGHF. It includes mid-term interactions performed in the modal representation phase and post-term interactions in the modal fusion phase. This approach allows the model to fully perceive various modalities' potential representational sentiment information, which helps us improve the fusion and prediction results. Although previous studies have shown that text modality is the most critical [9, 12], we still believe that the information implied by any modality should be considered in the MSA task. Specifically, MGHF employs a flexible strategy for modality variability by using appropriate neural networks for different modalities. In the medium-term interaction learning phase, MGHF performs cross-modal attention interactions for acoustic modality, visual modality, and text modality, respectively, to obtain text-based acoustic representation and text-based visual representation. Several past studies [13] have pointed out that task-related information is not evenly distributed across modalities, with the text modality contributing much more than other modalities. There are also studies [8, 9] that would fuse the text-video and audio modalities as a ternary symmetric structure, which does not take into account the variability of the various modalities and thus fails to fuse them correctly. According to previous experience, in order to make the text modality occupy a higher weight than other modalities in the later fusion stage. We combined the text-based acoustic representation with the text representation, the text-based visual representation with the text representation, and the text-based acoustic representation with the text-based visual representation in a two-by-two combination. We also design gated recurrent hierarchical fusion networks that dynamically interact with learning information representations between modal combinations to complement the information between combinations. Our extensive experiments on the publicly available and popular datasets CMU-MOSI [14] and CMU-MOSEI [15] show that MGHF shows strong competitiveness over previous complex interaction and fusion baselines.

The contributions of this paper are summarized as follows:

- A gated cyclic hierarchical fusion network for multimodal sentiment analysis is proposed. It dynamically interacts with information representations between 3 different modal pairs. The gated cyclic hierarchical fusion network enables sufficient interaction between each modal pair, eliminates redundant information between modal pairs, and maximizes the retention of valid representations for modal prediction.
- Inspired by distribution matching, we consider the interactions within different modalities. In the modal representation acquisition stage, we make the nonverbal sequences to cross-modal attention with text sequences, which can capture potential representations within different modalities while making the modal representations closer to the real sentiment expressions.
- Experiments conducted on two publicly available multimodal datasets show that our model has significant advantages over previous advanced complex baselines.

## 2. Related Work

This section introduces multimodal sentiment analysis, as well as related work on multimodal representation learning and data fusion.

### 2.1. Multimodal Sentiment Analysis

Unlike traditional sentiment analysis, multimodal sentiment analysis often uses multiple sources (excerpted text, audio, video, and other information) to fully and accurately predict the speaker's sentiment orientation. Researchers have various ways to deal with MSA tasks, one of which is representative of the extraction of intramodal temporal information and the other is the extraction of intermodal interaction information. The former mainly uses neural networks such as the Long Short-Term Memory (LSTM) Network [16] for the extraction of modal contextual information [10, 17]. The latter can be further divided into early, late, and hybrid, depending on the fusion stage. Early fusion is the fusion approach used in the pre-extraction phase of the data. Rozgic et al. [18] used early fusion to connect multimodal representations as input to an inference model, which provides a novel idea for modal fusion. Zadeh et al. [19] designed a memory fusion network (MFN) using multiview sequential learning, which explicitly illustrates two interactions in the neural architecture. The post-fusion approach performs a series of necessary processing within the modality and intermodal data fusion in the final stage. Liu et al. [20] proposed a low-rank multimodal fusion approach to reduce the computational complexity by using low-rank tensor fusion to improve efficiency. Other researchers have used hybrid fusion to improve the performance of MSA tasks. Dai et al. [21] used a simple but very effective hybrid modal fusion approach using weakly supervised multitask learning to improve the generalization performance of the dataset.

We differ fundamentally from previous work in that. First, there is a modal divide between different modalities, and using only the same neural network does not seem to yield useful information. Instead of considering a piece of single contextual information, we use the most appropriate strategy based on the modal sequence characteristics. After obtaining the initial representations, unlike in previous work, our interaction fusion does not only occur in the final stage. Useful potential information can be induced from the companion representations through the intermediate interaction stage. Similarly, the post-interaction stage of the modality is used to better retain information useful for prediction and eliminate redundant information. It is worth noting that instead of the traditional approach of treating text, audio, and video equally, we flexibly utilize the information useful to the task for each modality based on the contribution of the modality.

### 2.2. Representation Learning and Data Fusion

Representation learning methods can also be applied to multimodal sentiment analysis and have achieved significant results. Wang et al. [22] proposed a recursive attentional change embedding network to generate multimodal shifts. Hazarika et al. [10] proposed a way to learn multimodal invariant and specific representations while combining four different losses to evaluate the performance of the model. Yu et al. [11] proposed self-supervised multitask learning to learn modality-specific representations and introduced a single-peak annotation generation module to assist the main task channel. In the context of sentiment analysis, multimodal fusion is essential because sentiment cues are usually distributed over different modalities [23]. Xiangbo et al. [24] proposed an extended-squeezed-excitation fusion network (ESE-FN) that fuses multimodal features in the modal and channel directions. The network learns extended-squeezed-excitation (ESE) caveats in the modal and channel directions to effectively solve the elderly activity recognition problem. Shu et al. [25] proposed a new weakly shared deep transport network (DTN) for converting cross-domain information from text to images. This provides ideas for interconversion across modalities. Based on this, Tang et al. [26] proposed a new generalized deep transmission network (DTN) for the transmission of information across heterogeneous, textual, and visual domains by establishing parameter sharing and representation sharing layers.

In view of this, our model is based on the late fusion of representation learning. Unlike previous studies, we learn representations across intramodal interactions while employing different combinations of modal interactions to obtain intermodal representations.

## 3. Materials and Methods

In this section, we will detail the main components of our model and their specific roles.

### 3.1. Task Setup

Multimodal data sequences in sentiment analysis consist of three main modalities which are the text modality (*t*), acoustic modality (*a*), and visual modality (*v*), respectively. The goal of multimodal sentiment analysis (MSA) is to predict the speaker's emotional polarity from a segment of discourse, which is also the input to the model in this paper. First, given the input discourse *U*_*s*∈{*t*, *a*, *v*\}_, this paper uses *U*_*v*_ to denote visual modal information, *U*_*a*_ to denote acoustic modal information, and *U*_*t*_ to denote textual modal information. Here, *a* ∈ *R*^*T*_*a*_×*d*_*a*_^, *t* ∈ *R*^*T*_*t*_×*d*_*t*_^, *v* ∈ *R*^*T*_*v*_×*d*_*v*_^, and *T*_*s*∈\{*t*, *a*, *v*\}_ denote the sequence length of a discourse, and *d*_*s*∈\{*t*, *a*, *v*\}_ denote the dimensionality of the respective features.

### 3.2. Overall Architecture

In this paper, our multimodal sentiment analysis architecture consists of three primary and flexible modules as shown in Figure 2. They are the feature extraction module for each modality, the (acoustic-text/visual-text) cross-attention module, and the gated recurrent hierarchical fusion network module. For the text channel, we use pretrained BERT for its high-dimensional semantic extraction. For the acoustic and visual channels, we first feed the initial sequence into a 1D temporal convolution to obtain enough perceptual and temporal information. The obtained (acoustic/visual) representations are then learned cross-modally with textual representations, which can induce potential representational information for both acoustic and visual modalities, synergistic to the overall effective orientation. Notably, this cross-modal matching has been prominent in recent cross-modal learning approaches [27, 28]. Afterward, we feed the output of the two cross-modal attention (text-based acoustic representation and text-based visual representation) and the extracted textual modal representation into a gated recurrent hierarchical fusion network, which eliminates redundant modal information to obtain the final information for prediction. Of course, some of the modules in our model are flexible and can be reconfigured with any suitable baseline to accomplish different types of tasks.

### 3.3. Modality Representation

The acquisition of representation for our model is divided into three channels, namely, text channel, video channel, and audio channel. In the following, we describe the essential details of the model acquisition of representations.

#### 3.3.1. Text Channel

For the text channel, we fine-tuned the pretrained model BERT [29] used as an extractor of text features, consisting of a 12-layer stacked transformer. The input text is preprocessed and fed to BERT for embedding by adding two special tags CLS and SEP. Consistent with recent work, the first word vector of the last layer is chosen in this paper as the average representation of the representation in the final 768-dimensional implicit state [30].

(1) $$\begin{array}{c} t_{i}=\left\{\left[CLS\right],w_{1},w_{2},\ldots ,w_{n},\left[\text{SEP}\right]\right\},\\ f_{t}=\text{BERT}\left(t_{i},\theta_{t}^{\text{bert }}\right)\in R^{d_{t}},\;i\in \left[1,n\right]. \end{array}$$

Here, *t* represents the initial sequence of text and *θ*_*t*_^bert ^ represents the hyperparameters of the BERT pretrained model.

#### 3.3.2. Audio and Video Channels

For the audio and video channels, we designed two independent modal characterization modules for the nonverbal sequences, and they function before fusion. We followed previous work [11] and processed the raw data using a pretrained toolkit to obtain the initial vector features.

*Temporal Convolutions*. First, to make our modalities sufficiently perceptible, we pass the input sequence through a one-dimensional temporal convolution layer.
  (2) $$\begin{array}{c} U_{m}^{*}=\text{Conv}1\;D\left(U_{m},k_{m}\right)\in R^{T_{m}\times d}, \end{array}$$
where Conv1D(•) is the one-dimensional temporal convolution function, *k*_*m*_ is the size of the convolution kernel used by the modality m, *U*_*m*_ is the input sequence of modality *m*, *d* is the common dimension, and *T*_*m*_ denotes the discourse length of modality *m*; here, *m* ∈\{*a*, *v*\}.
*Positional Embedding*. To equip the sequences with temporal information, following Vaswani et al. [31], the position embedding (PE) is bracketed to *U*_*m*_^*∗*^ as follows:
  (3) $$\begin{array}{c} U_{m}^{{*}^{\prime }}=U_{m}^{*}+\text{PE}\left(T_{m},d\right), \end{array}$$
where PE(*T*_*m*_, *d*) ∈ *R*^*T*_*m*_×*d*^, the purpose is to compute the embedding for each position index. PE(•) represents the position embedding function, *m* ∈{*a*, *v*}.
*Cross-Attention Transformers*. We then perform cross-modal cross-attention on the resulting sequences, which induces potential representational information for both acoustic and visual modalities that are synergistic to the overall practical orientation. It is worth noting that our cross-modal attention occurs only between text and acoustic modalities and between text and visual modalities, which allows the text modality that contributes most to the task to be weighted higher than the other modalities and ensures the relative independence of the visual and acoustic channels. We justify this approach in Section 5.2.1.
  (4) $$\begin{array}{c} C\_{\text{Attention}}_{a-t}\left(Q,K,V\right)=\text{softmax}\left(\frac{Q_{t}K_{a}^{T}}{\sqrt{d_{h}}}\right)V_{a},\\ C\_{\text{Attention}}_{v-t}\left(Q,K,V\right)=\text{softmax}\left(\frac{Q_{t}K_{v}^{T}}{\sqrt{d_{h}}}\right)V_{v}, \end{array}$$
where *Q*_*t*_ represents the query vector for the text modality and *K*_*a*_, *V*_*a*_, *K*_*v*_, and *V*_*v*_ denote the key vectors and value vectors of the acoustic and visual modalities. softmax(•) represents the softmax function, *d*_*h*_ represents the dimensionality of the modality, and *T* represents transpose.

Transformer computes multiple parallel attentions, and the output of each attention is called a head. The *i*^*th*^ head is computed as

(5) $$\begin{array}{c} {\text{head}}_{m}^{i}=={\text{Attention}}_{m}\left(Q_{t}W_{i}^{Q_{t}},K_{m}W_{i}^{K_{m}},V_{m}W_{i}^{V_{m}}\right), \end{array}$$

where *W*_*i*_^*Q*_*t*_^ ∈ *R*^*d*_*t*_×*d*_*q*_^ is the weight matrix of *Q*_*t*_ when computing the head of the *i*^*th*^ text modality; *W*_*i*_^*K*_*m*_^ ∈ *R*^*d*_*m*_×*d*_*k*_^ is the weight matrix of *K*_*m*_ when computing the head of the *i*^*th*^*m* modality; and *W*_*i*_^*V*_*m*_^ ∈ *R*^*d*_*m*_×*d*_*v*_^ is the weight matrix of *V*_*m*_ when computing the head of the *i*^*th*^*m* modality, where *m* ∈\{*a*, *v*\}.

After that, we connect all heads of *m* modalities, which is denoted as *Y*_*m*_^*∗*^ as follows:

(6) $$\begin{array}{c} Y_{m}^{*}=\text{MultiHead}\left(Q_{t},K_{m},V_{m}\right)\\ =\text{Concat}\left({\text{head}}_{m}^{1},{\text{head}}_{m}^{2},\ldots ,{\text{head}}_{m}^{n}\right)W_{m}^{o}, \end{array}$$

where *W*_*m*_^*O*^ is the weight matrix multiplied after the splicing the head of *m* modalities and n denotes the number of self-attention heads we use. Here, we have *n* = 10, Concat(•) is the splicing operation, *m* ∈\{*a*, *v*\}.

Thus, the text-based acoustic representation *f*_*a*_*t*__ and the text-based visual representation *f*_*v*_*t*__ can be obtained.

(7) $$\begin{array}{c} f_{a_{t}}=\text{MultiHead}\left(Y_{a}^{*};\theta_{a}^{c-att}\right),\\ f_{v_{t}}=\text{MultiHead}\left(Y_{v}^{*},\theta_{v}^{c-att}\right), \end{array}$$

where *θ*_*a*_^*att*^={*W*_*a*_^*Q*^, *W*_*a*_^*K*^, *W*_*a*_^*V*^, *W*_*a*_^*O*^} and *θ*_*v*_^*att*^={*W*_*v*_^*Q*^, *W*_*v*_^*K*^, *W*_*v*_^*V*^, *W*_*v*_^*O*^} represent the main hyperparameters required for the cross-attention module.

### 3.4. Gated Cyclic Hierarchical Fusion Networks

In previous studies [10, 11], after obtaining valid representations, most of the modal representations are simply spliced directly for final prediction. This can inadvertently add redundant information to them. To allow the redundant information in the representations to be effectively removed, we designed a gated recurrent fusion network (see Figure 3). This module is flexible and can be paired with other benchmarks to enhance the effect. Of course, we also verified the effectiveness of the hierarchical fusion network.

We used the text-based acoustic representation *f*_*a*_*t*__ and text-based visual representation *f*_*v*_*t*__ as well as text representation f_t_ as inputs to the gated recurrent hierarchical network. Previous experience [9, 12] has shown that the text modality contributes much more to the task than the other modalities. Given this, we combined the text-based visual representation, the text-based acoustic representation, and the text representation in two combinations to ensure that the text modality accounts for a high weight, which would result in three combinations of representations.

(8) $$\begin{array}{c} f_{a_{t}⊕t}=\text{Concat}\left(f_{t},f_{a_{t}}\right),\\ f_{v_{t}⊕t}=\text{Concat}\left(f_{t},f_{v_{t}}\right),\\ f_{a_{t}⊕v_{t}}=\text{Concat}\left(f_{a_{t}},f_{v_{t}}\right). \end{array}$$

where Concat(•) denotes the combination operation, *f*_*a*_*t*_⊕*t*_ denotes the combination of text-based acoustic representation with text, *f*_*v*_*t*_⊕*t*_ denotes the combination of text-based visual representation with text, and *f*_*a*_*t*_⊕*v*_*t*__ denotes the combination of text-based acoustic representation with text-based visual representation.

After obtaining the specified three combinations, we fed them into a bi-directional gated recurrent network (Bi-GRU). The purpose of doing so is to allow the information between different modalities to be fully perceived and to effectively remove redundant and irrelevant information from the representations through the gating mechanism. We also employ a bi-directional long and short memory (Bi-LSTM) network. By comparison, we found that the former has more straightforward parameters and faster training speed, and its results are comparable.

(9) $$\begin{array}{c} f_{t-a}=Bi_{-}GRU\left(f_{a_{t}⊕t},\theta^{gru}\right),\\ f_{t-v}=Bi_{-}GRU\left(f_{v_{t}⊕t},\theta^{gru}\right),\\ f_{a-v}=Bi_{-}GRU\left(f_{a_{t}⊕v_{t}},\theta^{gru}\right), \end{array}$$

where *Bi*_−_*GRU*(•) represents the bi-directional gated recurrent cell network and *θ*^*gru*^ represents the hyperparameters of the gated recurrent cell network.

After that, we combine the outputs of the gated cyclic hierarchical fusion networks and feed them into the fully connected layer for the final prediction.

(10) $$\begin{array}{c} f_{s}=\text{concat}\left(f_{t-a},f_{t-v},f_{a-v}\right),\\ f_{s}^{*}=\text{ReLU}\left(W_{l1}^{sT}⊗f_{s}+b_{l1}^{s}\right), \end{array}$$

where *W*_*l*1_^*s*^ ∈ *R*^(*d*_*t*_+*d*_*a*_+*d*_*v*_)×*d*_*s*_^ and ReLU are the relu activation functions and ⊗ represents the elemental product.

 Finally,*f*_*s*_^*∗*^is used as the final representation and for the prediction task.

(11) $$\begin{array}{c} y^{\prime }=\text{ReLU}\left(W_{l2}^{sT}⊗f_{s}^{*}+b_{l2}^{s}\right), \end{array}$$

where *W*_*l*2_^*s*^ ∈ *R*^*d*_*s*_×1^.

## 4. Experiment

In this section, we will detail the specifics of our experiments.

### 4.1. Datasets

*CMU-MOSI* [14]. The Multimodal Sentiment Intensity Corpus dataset is a collection of 2199 viewpoint video clips. This dataset is a popular benchmark for multimodal sentiment analysis. Each opinion video is annotated with sentiment in the range of [−3, 3]. The dataset is strictly labelled using tags for subjectivity, emotional intensity, per-frame, per-viewpoint annotated visual features, and per-millisecond annotated audio features.

*CMU-MOSEI* [15]. The multimodal Opinion Sentiment and Sentiment Intensity dataset is the largest multimodal sentiment analysis and recognition dataset. The dataset is an improved version of the CMU-MOSEI dataset. MOSEI contains more than 23,500 sentence expression videos from more than 1,000 online YouTube speakers. The dataset is gender-balanced. All sentences were randomly selected from different videos of topics and monologues. Videos were transcribed and correctly punctuated. We give the detailed dataset settings in the experiments (see Table 1).

### 4.2. Modality Processing

To ensure fair competition with other baselines, we follow previous work [11] and treat the three modalities as a typical tensor described as follows:

 
*Text Modality*. Most previous studies have used glove [32] as a source of word embedding and achieved good results. Considering the strong performance of pretrained models, we prefer to use the pretrained language model BERT [29]. For a fair and objective comparison, we adopted the latter as the processing tool for our text modality.
 
*Audio Modality*. For audio data, the acoustic analysis framework COVAREP [33] was used to extract up to 12 Mel-frequency cepstral coefficients, pitch, turbid/apparent segmentation features, and so on. All features are related to mood and intonation. It is worth noting that acoustic features are processed to align with the text features.
 
*Video Modality.* Video modality raw features are used to extract facial expression features using Facet (https://imotions.com/platform/), which includes facial action units and facial poses based on the Facial Action Coding System (FACS) [34]. The process is repeated for each sampled frame within the vocalized video sequence.

Eventually, we align the initial modalities with the text for the alignment operation. This will allow our experiments to proceed appropriately and ensure fair experimental comparison results.

### 4.3. Evaluation Metrics

Again, to be fair, we split the MSA task into a regression task and a classification task. This paper will have five valuation metrics, which are: secondary precision (ACC-2) and F1-score. Mean Absolute Error (MAE): it directly calculates the error between the prediction and the authentic number labels. Level 7 Precision (ACC-7) and Pearson Correlation (Corr) measure the standard deviation from the human-annotated actual value. It is worth noting that the secondary precision and F1 scores were divided into two groups: negative and non-negative feelings (including neutral feelings), and negative and positive feelings, respectively. In addition to the value of MAE, higher scores imply better results.

### 4.4. Baseline

We compared the performance of MGHF with several multimodal fusion frameworks, including state-of-the-art models, as follows.

#### 4.4.1. Previous Models

- *TFN.* Tensor fusion network [8] is based on Cartesian product to calculate the tensor of each modality for capturing the interaction information of unimodal, bimodal, and three modalities.
- *LMF*. Low-order multimodal fusion [20] is an improvement of the tensor fusion network (TFN) to reduce the computational complexity and improve the efficiency by using low-order tensor fusion.
- *MFM*. Multimodal Factorization Model [35] demonstrates flexible generation capability by adjusting independent factors and reconstructs missing modes.
- *MULT*. Multimodal Transformer (MULT) [9] extends the multimodal converter architecture using directed pairwise cross-attention, which converts one modality to another using directed pairwise cross-attention.
- *ICCN*. Interaction Canonical Correlation Network (ICCN) [13] learns correlations between text, audio, and video through Deep Typical Correlation Analysis (DCCA).
- *MISA*. Learning Modality-Invariant and Modality-Specific Representations (MISA) [10] combines a combination of distribution similarity, orthogonal loss, reconstruction loss, and task prediction loss for learning the representation of different modalities and the representation of fused modalities.
- *MAG-BERT* [36]. A multimodal adaptation gate was designed for the BERT alignment gate and inserted into the general BERT model to optimize the fusion process.

#### 4.4.2. State-of-the-Art

For sentiment analysis tasks, the results of Self-MM [11], a self-supervised multitask learning framework, on both MOSI and MOSEI datasets represent state-of-the-art (SOTA) models. Self-MM assigns a single-peaked training task with automatically generated labels to each modality, allowing multimodal sentiment analysis tasks to be performed in a multitask context.

## 5. Results and Discussion

In this section, the experimental results of the model are analysed and discussed in detail.

### 5.1. Quantitative Results

We compared the MGHF with currently popular benchmarks, including the state-of-the-art (SOTA) model (see Tables 2 and 3). For a fair comparison, we divided the models into two categories depending on the data setup, aligned and unaligned. In our experiments, first, compared with the aligned advanced models, our models all achieved similar or even surpassed results. In addition, our models achieve significant gains on all indicators of the regression as well as on some of the categorical indicators compared to the unaligned models. In addition, we reproduce two strong baselines, MISA and self-mm, under the same conditions. We find that MGHF outperforms them on most indicators. On the MOSI dataset, MGHF achieves competitive scores on both classification tasks. On the regression task, MGHF also improves the SOTA model by various degrees. Our model also outperforms some complex fusion mechanisms, such as TFN and LFN. The above results show that our model can be applied to different data scenarios and achieve significant improvements. We visualized some of the metrics, which can help us visualize how the model is performing (see Figure 4).

### 5.2. Ablation Study

We set up ablation experiments to verify the performance of our model, which is divided into the following main parts.

#### 5.2.1. Representational Interaction

First, for cross-modal attention interactions, we conducted the following experiments. The first group was performed for the interaction between two modalities, and we did not consider acoustic-based text features and visual-based text features because this would make the text modality so heavily dominated that modal independence would be reduced or even disappear. The cross-modal attention between nonverbal sequences is hardly satisfactory, probably due to the characteristics of nonverbal sequence data. Acoustic, visual, and textual cross-modal attention seems to play an important role, which is consistent with previous studies [9, 12]. The second set of experiments was conducted after combining the cross-modal interaction representations obtained in the first set, which could help us elucidate whose combination of cross-modal interactions is more beneficial for the MSA task. In Table 4, it seems apparent that the combination of text-based acoustic and text-based visual representations performs the best. We believe this is partly because the text modality enhances the complementary acoustic and visual information, providing additional cues for semantic and affective disambiguation [37], and partly because it preserves the independence of the acoustic and visual modalities. We visualized this part of the experimental index scores for ten randomly selected samples from the MOSI test set (see Figure 5), and similar results were observed on MOSEI.

#### 5.2.2. Gated Recurrent Hierarchical Fusion Network Effectiveness

To verify the reliability of our proposed gated cyclic hierarchical fusion network, we will perform the multimodal sentiment analysis task under the same conditions without this fusion strategy. For visual comparison, two representative metrics from the classification and regression tasks are selected for evaluation, while the evaluation results are visualized. It is worth noting that among these metrics, higher scores imply better performance, except for the MAE metric. The results are shown in (Figure 6). Specifically, the gating mechanism effectively removes the redundant information contained in the previous stage. This not only implies that the representations obtained by the model in the prediction stage are inclusive of the potential representations of each modality but also helps us clarify the need for representation interaction learning at a later stage.

In addition, we also conduct ablation experiments of the fusion strategy (as shown in Table 5). In this experiment, we do not combine the resulting text-based visual modality, text-based acoustic modality, and text modality. The settings are marked as “a” in Figure 7 and MGHF_*w/o(pc)* in Table 5. At the same time, we replace Bi-GRU in the fusion network with Bi-LSTM neural network. This setting is marked as “b” in Figure 7 and MGHF_*LSTM* in Table 5. As mentioned before (Section 3.4), only in this experiment does Bi-GRU achieves comparable or even better performance on some metrics.

 As shown in the previous section (Section5.2.1) the combined contribution of text-based sound representations *f*_*a*_*t*__ and text-based visual representations*f*_*v*_*t*__ is the highest. We used these two representations combined with the initial representations *f*_*a*_, *f*_*v*_, and *f*_*t*_ to evaluate which set performs best for the hierarchical fusion network (see Table 6). It is easy to see that the combination of *f*_*a*_*t*__ and *f*_*v*_*t*__ with the textual representation *f*_*t*_, which is the input to our gated recurrent hierarchical fusion network, performs best.

## 6. Conclusions

In this paper, we propose a complete solution for multimodal sentiment analysis, MGHF, which differs in two main parts: modal representation and modal fusion. By using distribution matching in the representation learning phase, the neighbouring modalities are made to contain potential representations of the companion modalities to achieve modal information interaction in time series. Meanwhile, we design a gated recurrent hierarchical fusion network in the fusion phase through the intermodal representation interactions performed in the later fusion phase. It eliminates redundant modal representations and retains those valid for prediction in the final stage, making the prediction results closer to the actual scores. We show that our model is intensely competitive with previous complex baselines through extensive experiments on two publicly available datasets.

## Figures and Tables

**Figure 1:** The combination of different modal pairs and sentiment prediction results.

**Figure 2:** MGHF: cross-modal attention with hierarchical recurrent fusion network.

**Figure 3:** Gated cyclic hierarchical fusion network.

**Figure 4:** Comparison of the performance of each baseline model. (a) F1-score. (b) Acc-2.

**Figure 5:** Visualization of different cross-modal interactions and their combined performance. (a) Corr. (b) MAE (the lower the better).

**Figure 6:** Gated cyclic hierarchical fusion network performance visualization.

**Figure 7:** Ablation research in fusion strategies.

**Table 1:** MOSI and MOSEI dataset size settings.

Dataset	MOSI	MOSEI
Train	1284	16326
Valid	229	4659
Test	686	1871
All	2199	22856

**Table 2:** Results on MOSI. Note: (B) Means the language features are based on BERT; model with ^*∗*^ represents the best results for recurrence under the same conditions. ○ is from[10], and ◇ is from [11]. In indicators Acc-2 and F1-score, the left side of “/” is calculated for negative and non-negative sentiment, while the right side of “/” is calculated for negative and positive sentiment.

Models	MOSI					Data setting
	MAE (↓)	Corr (↑)	Acc-7 (↑)	Acc-2 (↑)	F1-score (↑)	
TFN (B)^○^	0.901	0.698	34.9	−/80.8	−/80.7	Unaligned
LMF (B)^○^	0.917	0.695	33.2	−/82.5	−/82.4	Unaligned
MFM (B)^○^	0.877	0.706	35.4	−/81.7	−/81.6	Aligned
MULT^*∗*^	0.918	0.680	36.47	77.93/79.3	77.91/79.34	Aligned
ICCN (B)^◇^	0.860	0.710	39.0	−/83.0	−/83.0	Unaligned
MISA (B)^◇^	0.783	0.761	42.3	81.8/83.4	81.7/83.6	Aligned
MAG-BERT (B)^◇^	0.731	0.789	—	82.54/84.3	82.59/84.3	Aligned
Self-MM (B)^◇^	0.713	0.798	—	84.42/85.95	84.42/85.95	Unaligned
MISA (B)^*∗*^	0.759	0.787	42.57	81.05/82.93	81.03/82.97	Aligned
Self-MM (B)^*∗*^	0.718	0.796	45.77	83.09/84.09	83.10/84.96	Aligned
MGHF (B)	0.709	0.802	45.19	83.38/85.21	83.32/85.21	Aligned

**Table 3:** Results on MOSEI. Note: (B) Means the language features are based on BERT; model with ^*∗*^ represents the best results for recurrence under the same conditions. ○ is from [10], and ◇ is from [11]. In indicators Acc-2 and F1-score, the left side of “/” is calculated for negative and non-negative sentiment, while the right side of “/” is calculated for negative and positive sentiment.

Models	MOSEI					Data setting
	MAE (↓)	Corr (↑)	Acc-7 (↑)	Acc-2 (↑)	F1-score (↑)	
TFN (B)^○^	0.593	0.700	50.2	−/82.5	−/82.1	Unaligned
LMF (B)^○^	0.623	0.677	48.0	−/82.0	−/82.1	Unaligned
MFM (B)^○^	0.568	0.717	51.3	−/84.4	−/84.3	Aligned
MULT^○^	0.580	0.703	51.8	−/82.5	−/82.3	Aligned
ICCN (B)^○^	0.565	0.713	51.6	−/84.2	−/84.2	Unaligned
MISA (B)^◇^	0.555	0.756	52.2	83.6/85.5	83.8/85.3	Aligned
MAG-BERT (B)^◇^	0.539	0.753	—	83.79/85.23	83.74/85.08	Aligned
Self-MM (B)^◇^	0.530	0.765	—	82.81/85.17	82.53/85.30	Unaligned
MISA (B)^*∗*^	0.558	0.748	51.45	82.14/85.09	82.44/84.94	Aligned
Self-MM (B)^*∗*^	0.534	0.764	53.32	84.37/85.28	84.42/85.06	Aligned
MGHF (B)	0.528	0.767	53.70	85.25/85.30	85.09/84.86	Aligned

**Table 4:** Performance tables for different cross-modal notes on MOSI and MOSEI datasets.

Task	MOSI				MOSEI			
	MAE (↓)	Corr (↑)	Acc-2 (↑)	F1-score (↑)	MAE (↓)	Corr (↑)	Acc-2 (↑)	F1-score (↑)
*f*_*a*_*v*__	1.442	0.210	53.81	46.48/	1.315	0.197	60.13/61.25	60.48/59.38
*f*_*v*_*a*__	1.321	0.233	62.33	57.85/58.94	1.244	0.182	58.48/59.47	61.63/61.48
*f*_*a*_*t*__	0.896	0.393	68.52	64.44/65.38	0.815	0.213	64.15/63.18	64.85/64.25
*f*_*v*_*t*__	0.901	0.384	71.49	69.12/67.20	0.843	0.241	63.48/63.14	63.54/63.89
*f*_*v*_*t*__+*f*_*a*_*v*__	0.976	0.223	73.62/71.40	71.04/64.31	0.821	0.213	61.84/62.37	61.23/61.66
*f*_*a*_*t*__+*f*_*v*_*a*__	0.957	0.381	74.22/72.67	71.04/65.86	0.784	0.230	63.24/62.56	61.05/60.72
*f*_*a*_*t*__+*f*_*v*_*t*__	0.819	0.486	76.80/76.01	75.72/74.84	0.763	0.361	72.18/72.56	74.37/74.03

**Table 5:** Ablation study results of fusion strategies on MOSI and MOSEI datasets.

Task	MOSI				MOSEI				
	MAE (↓)	Corr (↑)	Acc-2 (↑)	F1-score (↑)	MAE (↓)	Corr (↑)	Acc-2 (↑)	F1-score (↑)	
MGHF_*w/o(pc)*	0.714	0.793	82.88	82.63	0.538	0.758	84.27		84.48
MGHF_*LSTM*	0.712	0.800	83.27	82.94	0.530	0.767	85.22		84.89
MGHF_*original*	0.709	0.802	83.38	83.32	0.528	0.767	85.25		85.09

**Table 6:** Effect of inputs on prediction results for different gated cyclic hierarchical fusion networks on MOSI and MOSEI datasets.

Input	MOSI				MOSEI			
	MAE (↓)	Corr (↑)	Acc-2 (↑)	F1-score (↑)	MAE (↓)	Corr (↑)	Acc-2 (↑)	F1-score (↑)
*f*_*a*_+*f*_*a*_*t*__+*f*_*v*_*t*__	0.887	0.641	78.56	78.42	0.699	0.548	80.92	80.33
*f*_*v*_+*f*_*a*_*t*__+*f*_*v*_*t*__	0.852	0.728	80.74	80.57	0.644	0.615	82.14	82.06
*f*_*t*_+*f*_*a*_*t*__+*f*_*v*_*t*__	0.709	0.802	83.38	83.32	0.528	0.767	85.25	85.09

## Data Availability

The data used to support the findings of this study are available on the following address. Dataset Address: https://immortal.multicomp.cs.cmu.edu/raw_datasets/processed_data/.
